RETRACTED

# Processing Decision Tree Data Using Internet of Things (IoT) and Artificial Intelligence Technologies with Special Reference to Medical Application

**DOI:** 10.1155/2022/8626234

**Published:** 2022-06-28

**Authors:** Latefa Hamad Al Fryan, Mahasin Ibrahim Shomo, Malik Bader Alazzam, Md Adnan Rahman

**Affiliations:** ^1^Educational Technology, Faculty of Education, Princess Nourah University, Saudi Arabia; ^2^Applied College Education (Curriculum & Instruction), Princess Nourah University, Saudi Arabia; ^3^Information Technology College, Ajloun National University, Jordan; ^4^Adjunct Faculty at Green Business School, Green University of Bangladesh, Dhaka, Bangladesh

## Abstract

Alternative methods are available for a wide range of medical conditions. Idealistically, doctors would have a tool that would analyse their patients' symptoms and suggest the most accurate diagnosis and treatment plan. Artificial intelligence uses decision trees to predict and classify large datasets. A decision tree is a versatile prediction model. Its main purpose is to learn from observations and logic. Rule-based prediction systems represent and categorize events. We discuss the basic properties of decision trees and successful medical alternatives to the classic induction strategy. The study reviews some of the most important medical applications of decision trees (classification). We show researchers and managers how to accurately assess hospital and epidemic management behaviour. Additionally, we discuss decision trees and their applications. The results showed the effectiveness of decision trees in processing medical data by using internet of things (IoT) and artificial intelligence technologies in medical applications. Accordingly, the researchers recommend the use of these technologies in other fields of studies.

## 1. Introduction

Industry research was an early adopter of data mining. Inductive processes based on decision trees developed in decision theory were also introduced at the same time. Specialized technologies such as learning (machine learning) and pattern recognition have emerged as a result of the advancement of computing (pattern recognition). Since the development of modern computers, a decision tree (DT) is a representation of a multivariate function that can be used in everyday life. Sonquist-Morgan (1964) seminal work on the AID (Automatic Interaction Detection) [1] software sparked interest in the practical use of DTs, which arose from the needs of the social sciences. As a result, the DTs have progressed from being merely an illustrative representation in decision-making courses to becoming a practical and easy-to-use tool. “Classification Stone's and regression trees” [2, 3] completed these advancements. It was proposed that a practical method of induction be used to build DTs recursively. CART is the acronym for this. Creating the ID3 (Iterative Dichotomiser 3) algorithm creates trees based on information entropy. The author improved it and dubbed it C4.5 (1993) [4]. These methods are capable of correcting the flaws in the DT used in classical decision theory. Some patient data may be missing in medical practice due to broken or missing equipment, the inability to perform the test, or other factors. On the other hand, by using only one training sample, this results in a single DT. If there is a variable missing from the patient's information, this is the case. The doctor will want to have DT and use it before deciding so that he does not miss out on the benefits of using DT as an auxiliary tool. On the other hand, the user would value the ability to analyse multiple DTs and the fact that the DT's predictive efficiency would improve as a result of the new information. These algorithms largely compensate for these flaws. Cremilleux-Robert (1997) [5] created a framework for using DTs in medicine. [6] criticised this, citing the limitations of this technique when used with medical students. With 2637 cases used DT's to consider in the treatment of fractures. Contribution of study identifies and predicts massive datasets, and artificial intelligence used decision trees. Some of the most important medical uses of decision trees are discussed in the research (classification). The goal of this research was to find the best induction method.

RETRACTED

## 2. Data Mining and Classification Trees

### 2.1. Data Mining

Data mining (DM) necessitates operations that must be analysed by a statistician, or someone who understands both the concepts and how to interpret the data when changes occur. One of the issues raised by the dialectic of the exploratory-inferential statistics pair is this. The first performs data analysis, and data mining is used in this process. The second tool allows you to conclude data generated by a phenomenon. As a result, DM necessitates iteration between the fields of computing and statistics and the areas where it is applied by experts, such as doctors in medicine [7].

Because of its features, transparency, and low cost of data storage, the DM became increasingly popular. This is usually only classified when it comes to its role in the study of large databases, and it falls under the heading of “Knowledge Discovery in Databases.” It is more accurate to define DM as a process that extracts essential information from large databases without requiring any prior knowledge to make decisions and learn about the phenomenon.

RETRACTED

DM should be viewed as a multidisciplinary field that connects procedures, methods, models, and techniques from statistics, pattern recognition, and machine learning, among other fields. The presence of variety in the DM facilitates the selection of tools, which is critical. Inductions lead to inferences, which lead to general models from a concrete example that generates a sample or population. By analysing known cases, the goal is to learn to classify the items. The importance of such a process in medicine, for example, is obvious in identifying the best therapies for various ailments as shown in Figure 1.

The potential of the DM to work with the size of the databases to be analysed is of great importance. As there are several possible sources of data, the application of the DM requires the so-called “Data Warehouse.” This is a relational database management system. It is used to extract archived operational data, resolve inconsistencies between different data formats, and integrate them. Once processed and accumulated in the Data Warehouse, the data is not updated or altered and simply loaded or accessed [8]. Let us think about patient records and the information that can be collected about them from databases in various health centres. The need to use a Data Warehouse that collects data from various databases, classifies them, and cleans up inconsistencies is exemplified.

### 2.2. Decision Trees

Decision trees provide a very powerful classification tool. Its use in data management makes it popular, given the possibilities it offers and the ease with which its results are understood by any user. The tree itself, when obtained, determines a decision rule. This technique allows:

Sample.

- *Segmentation*. Establish which groups are important to classify a certain item. *Classification*. Assign items to one of the groups in which a list is partitioned
- *Prediction*. Establish rules to make predictions of certain events. *Reduction of the Dimension of the Data*. Identify which data are important to make models of a phenomenon
- *Identification-Interrelation*. Identify which variables and relationships are important for certain groups identified from analysing the data
- *Recoding*. Discretize variables or establish qualitative criteria losing the least possible amount of relevant information

The need to make new investments is constant in the health sector, especially in the public sector where decisions involve politicians. In particular, these investments are associated with the acquisition of new instruments, which can be expensive, expendable material, or extensions-repairs. For them, decisions involve the demand for large sums of money from financial sources. These decisions have repercussions with a delay in the service quality, but it immediately affects the finances and the long-term goals previously set. Investments are strategic decisions and are associated with a high degree of uncertainty [9]. All these investment decisions are supported by expert predictions. In investment analysis, the use of the concept of expected value is popular, and we can use it in the construction of decision trees.

RETRACTED

The expected value represents the long-term average to be obtained under the principle of repeated sampling. It is assumed that a probability measure *P*(*X*) allows establishing several scenarios whose result is characterized by a realization *X* that can take *k* possible values *x*_1_,…, *x*_*k*_. The expected value *E*(*X*) is as follows

(1) $$\begin{array}{c} E\left(X\right)=\overset{k}{\underset{i=1}{\sum }}x_{i}P\left(X=x_{i}\right). \end{array}$$

The decision tree will allow us to represent and analyse the result of the investment. Before purchasing new equipment, the management of a hospital has a decision tree. Each decision leads to one of the terminal nodes and is associated with a monetary and/or prestige cost. The probability of travelling each path is established by them. It is clear that if the purchase was not made, the service would not be provided with probability one and that if it were, the improvement would be provided with the same probability. In the first case, there is no monetary cost, but socially, the prestige of the health third will be affected.

In the evaluations, the reasoning present in the dynamic programming of “backward induction” is used: starting at a final node, it returns to the initial node. This decision tree is the one used in classical decision theory. These lead to poor algorithms for making inductions when the data is incomplete (missing) or with many errors (noisy data).

On the other hand, when evaluating a patient's symptoms, a doctor detects information through answering questions and rules out possible diseases that may afflict him. In her mind, she has a decision tree and reaches a conclusion, or several possible ones, by considering how plausible the path she follows based on her questions' answers. When evaluating a questionnaire or analysis, the doctor traces a path in a graph reaching a final node (leaf) [10]. Thus, a doctor's interest is to use the information collected and establish in which nodes the possible disorders are concentrated. Similarly, a researcher could analyse a health system to detect which care centres concentrate on certain properties, such as the level of efficiency, for example, see Figure 2.

RETRACTED

In many medical problems, it is interesting to design the tree described by its users to consider the performance of a health system, which can range from a national system to that of a hospital.

To make such trees, a sample is taken, the path followed by the interviewees is observed, and any campaign or development plan would focus on satisfying the quality interests expressed by the interviews. Some paths will be followed more frequently, allowing a statistical analysis to be made of how the interviewees, who are nothing more than clients, evaluate the system and its components. For example, if we consider the use of a specialized hospital such as a heart centre, several paths traveled before reaching it can be considered [11]. For example, the general medical path-proximity-confidence-speed-poor diagnosis can be more opposite than polyclinic-proximity-confidence-slowness-correct diagnosis to reach treatment in a heart centre. This would lead us to obtain that the largest part of those who attend the emergency room of the cardio centre are patients who go to the polyclinic and live near it. This may lead to the need to establish closer permanent cardiology services in the municipalities and/or provide specialized training to general practitioners.

In medicine, decision making is very important and systematic. Think of diagnostics, for example. In advanced institutions, there are systems known as “Decision support systems,” decision support systems, which are used to help the doctor to establish alternative decisions, which are efficient and reliable in complex situations. These systems are generally capable of automatically training themselves with new information and learning (Automatic Learning). For such tasks, decision trees are a convenient tool. Given their performance in many applications, the experts in the various areas taken regularly use them because their behaviour is transparent. The use of a tool that leads us to determine DT is highly recommended when:

- We study concepts of the attribute-value type
- The objective function is associated with an RV with discrete values
- Item descriptions are disjunctive
- The learning set *T* has errors and/or has missing values

A DA formalizes a problem mapping by determining connections between tree nodes where the population study process is expressed by determining subtrees and leaves. Each leaf or terminal node determines a class that determines the decision. Some nodes are called test nodes, and output is elaborated based on the analysis of the data that has entered it from the previous nodes with which it connects. In its practical uses, DT begins by analysing known cases. The items are divided into two subsets. One is used to determine the tree (training sample) and the other to evaluate the effectiveness of the DT (test sample). An attribute is set to represent the decision of interest (response variable (RV)). The problem is determined by fixing a set of attributes that can be represented as a vector $\overset{⟶}{X}\in {ℛ}^{k}$ for each item. Then, we can say that the training sample is *T* = {*x*_1_, *x*_2_, ⋯, *x*_*m*_}.

RETRACTED

Attributes can take discrete, continuous, or qualitative values. In the discrete case, each value determines a class. If the variable is continuous, intervals will be determined. Qualitative variables are discretized. At each step, the set of items is subdivided according to a certain criterion into two or more classes until reaching the set of final nodes [12]. The usual method of partitioning is done by determining hyperplane orthogonal to the selected attribute. Thus, the DT divides the space *ℛ*^*k*^ into hyperrectangles, and each one identifies a decision. There is *m* − 1 possible partitioning of *T*. A pruning criterion is used to determine when to stop the segmentation to make a partition. If the number of VS's is high, the DT will be very large, making it difficult to interpret.

In the case of continuous attributes, intervals can be determined using one of the following criteria

- *Intervals with the Same Amplitude*. The number of classes is fixed, and the intervals are determined
- *Intervals Determined by Percentiles*. The number of classes is finalized, and the intervals are determined, looking for them to contain the same approximate number of items

Following [4], we can fix the search for DT as follows:

- If there are *k* classes denoted {*C*_1_, *C*_2_, ⋯, *C*_*m*_}, and a training set, *T*, then

If *T* contains one or more objects belonging to a single class *C*_*j*_; then, the decision tree is a leaf identifying class *C*_*j*_.

(ii) If *T* contains no objects, the decision tree is a leaf determined from information other than *T*
(iii) If *T* contains objects that belong to a mixture of classes; then, a test is chosen, based on a single attribute, that has one or more mutually exclusive outcomes {*O*_1_, *O*_2_, ⋯, *O*_*n*_}
(iv) *T* is partitioned into subsets *T*_1_, *T*_2_, ⋯, *T*_*n*_, where *T*_*i*_ contains all the objects in *T* that have the outcome *O*_*i*_ of the chosen test

The same method is applied recursively to each subset of the training object.

Let *S* ⊂ *Ω*

(2) $$\begin{array}{c} \Omega =\text{study population}=U_{1\leq i\leq n}C_{i}. \end{array}$$

When selecting a sample, a signal is obtained about the belonging of an item to a class. If

(3) $$\begin{array}{c} f\left(j_{i},S\right)=\text{number of objects in }C_{i},P_{i}=\frac{f\left(j_{i},S\right)}{\left|S\right|}. \end{array}$$

Thinking in terms of information theory, this signal in terms of bits is −log_2_*f*(*j*_*i*_, *S*)/|*S*|. Considering *S*, the information expected from the signal is

(4) $$\begin{array}{c} \inf\left(S\right)=-\frac{\text{lo}{\text{g}}_{2}f\left(C_{j},S\right)}{\left|S\right|}. \end{array}$$

If we have a training sample

(5) $$\begin{array}{c} \inf\left(\text{T}\;|\;\Omega \right)=\overset{n}{\underset{i=1}{\sum }}\left(\frac{\left|T_{i}\right|}{\left|T\right|}\right)\inf\left(T_{i}\;|\;\Omega \right). \end{array}$$

We then have a series of measures of interest on the partition.

RETRACTED

We then have a series of measures of interest on the partition. We are interested in *g* (*Ω*) = info (*T*) − info_*Ω*_ (*T*) = gain in information by partitioning *T* according to *Ω*. If we partition *T* into *n* subsets, we have

(6) $$\begin{array}{c} \text{part}-\text{info }{\left(\Omega \right)}_{i}=\inf\left(T\;|\;\text{X}\right)=i=\overset{n}{\underset{i=1}{\sum }}\left(\frac{\left|T_{i}\right|}{\left|T\right|}\right)\text{lo}{\text{g}}_{2}\left(\frac{\left|T_{i}\right|}{\left|T\right|}\right). \end{array}$$

The partition generates information that is useful for classification, and a measure of the gain is *gr* (*Ω*) = *g*(*Ω*)/part − info (*Ω*)_*i*_ = impurity function.

This measures the mixing of a subset and partitions to decrease impurity. It seeks to maximize it. Ultimately, this carries the same meaning as the Gini index, used in economics, [7]. This function considers the probability of misclassifying an additional sample given the result obtained by using the training sample *T*.

A classification rule will assign a new item to a node seeking to minimize the misclassification rate.

So a DT is a graph determined from some method that models decision making using easily understood rules. The items grouped from the attributes (explanatory or segmentation variables, VS) are obtained by segmenting *T*. When determining a group, a study is made, preferably statistical, of the VR. The homogeneity of this attribute is performed to explain the effect of the VS's on the VR. From the VS's, the members of the groups are identified, and it is easier to predict the value of the VR. This is nothing more than a marketing problem with particular characteristics. Thus, if we interview the system's users, it faces several questions. Your answers establish movement from one node to another in the tree, and at the end, you have traced a path to a conclusion represented by one of the final nodes [13]. Thus, the interviewee is classified. In the diagnostic area, the path leads to evaluating a decision rule. The symptoms that lead to certain diseases and the elements that most frequently identify them can be particularized by analysing the final nodes. The doctor will be able, using them, to have a group of possible diagnoses on which he will develop alternative treatments for the patient's ailment. This is of particular importance in diseases with many symptoms that are common to others, such as dengue.

RETRACTED

In both cases presented, the interest is to determine a highly plausible tree. Also, in both, a certain decision-maker, faced with different conditions, has evaluations that determine the decision-making that leads to a terminal node. If the tree design from taking a sample is plausible, it will affect the decisions made using them.

### 2.3. Decision Trees and Neural Networks

Most of the problems we tackle doing exploratory statistics have clear connections to AI. However, statisticians and AI specialists often do not communicate effectively. The terms used by one and the other are different, although the methods used are similar or the same. In practice, the entire arsenal of statistical methods and tools is wasted by AI. New and generally theoretically inefficient methods are created to solve problems that have been obtained and seem to be found in simple statistics textbooks [14]. AI has focused on making efficient algorithms and not using efficient inferential models.

To illustrate the difference in concepts' denomination, we use the table presented by Lebart (1998), Table 1.

RN is generalizations of classical statistical models that apply sequential learning and successfully address transformations of the original variables to make predictions and overcome the problems posed to statisticians by nonlinear models characterizing complex phenomena. This is a black box where the algorithm uses inputs and provides outputs. The system is expected to learn by improving its predictions. The methods of constructing DT and RN are complementary [15]. Representation through DT is transparent to the doctor and any user, but this is not the case with RN.

On the other hand, the DT technique fails when there are many outliers, which does not happen with the RN. Also, if we use DT to learn, learning is slow, but RNs do it quickly. Hence, the success of combining both techniques. The proposals use an RN that they train and turn into DT at the end of the learning. If the learning is good, the determined DT is better than the DT used as input data for the RNs.

### 2.4. Evolutionary Algorithms

Another technique used contemporaneously to build DT is the evolutionary algorithms (EVOP). These are commonly used in optimization if there is no efficient heuristic algorithm. [6–15].

RETRACTED

The quality of the DT is measured by

(7) $$\begin{array}{c} \text{LFF}=\overset{k}{\underset{i=1}{\sum }}w_{i}\left(1-acc_{i}\right)+\overset{N}{\underset{i=1}{\sum }}c\left(w_{i}\right)+w_{u}+nu1, \end{array}$$

where *k* is the number of decision classes. *N* is the number of attribute nodes in the tree. *acc*_*i*_ is the accuracy of the classification of items of a decision class di. *w*_*i*_ is the importance given (weight) to classify the items in the decision class di. *c*(*w*_*i*_) is the cost of using the attribute in a node ti. *nu* is the number of nodes not used.  *w*_*u*_ is the weight of the presence of unused nodes in the tree.

A tree will be better if LFF is smaller. The EVOP searches for the tree with the minimum value of LFF.

## 3. Its Success in Some Applications in Medicine

DT's have been used in medical and community health studies for more than two decades. We will see some applications made using the tools discussed.

Letourneau et al. (1998) took a sample of two groups of nurses and developed a DT to guide the work of one of them. It was concluded that this was of great help when comparing the group's efficiency helped by the DT and the one that did not use it. Tsien et al. (2000) used data obtained in Edinburgh and established how DT could be helpful in rapid decision making when making predictions in Sheffield.

Jones (2001) studied the use of DT's to fix signals suggestive of drug side effects. The DT technique has been proposed in the hospital setting to improve alarm systems in intensive care units, see Tsien et al. (2000). Bonner (2001) conducted a similar study with the mentally ill.

### 3.1. Study of the Behaviour of the Total Success of Emergency Surgery Cases

A study of 285 cases admitted to the emergency room in hospitals of a health system was carried out. All of them had to undergo emergency surgery. The hospital conditions at the time of the intervention, the conditions under which it was carried out, and the total success of the same were analysed. Total success refers to the absence of postoperative complications. Deaths were not considered in the study, as shown in Table 2, Table 3, and Figure 3.

The study of information entropy (EI) was carried out. The entropy is *I*(*S*) = 0.8631.

So the most important thing for the success of an urgent intervention is the level of urgency. It is followed by the level of the surgeon's auxiliary staff. This must be analysed carefully, meaning that the surgeon's level is important (being good or average according to a previous evaluation). This reflects that surgeons are not especially distinguished in such cases but that the intervention depends a lot on the qualification of the auxiliary personnel (nurses, anesthesiologists, etc.).

RETRACTED

### 3.2. Evaluation of a Placebo Ointment in Patients with Psoriasis on Less than 10% of Their Body

Three hundred sixty people who have psoriasis underwent placebo treatment. The medication was an ointment that came in two colours, *A* = blue and red. The results were evaluated, obtaining the results in the following Table 4.

The classification tree appears in Figure 4. It is noted that those who selected the red ointment considered they obtained improvement in less than 4.5 weeks (29.44%) and those of the blue in dismay without improvement after 8.1 (34.44%). Those who used the blue ointment were first considered cured, not improved, and 35.55% were discharged.

### 3.3. Study of Hygienic Conditions and Efficiency in Surgical Hospitals

Six classified hospitals poorly valued by their patients were analysed. The interest was to classify them into unreliable and reliable. The results of the audits led to Table 5 and Table 6.

Calculating the entropy of information (EI), we have that the entropy of primary care is *I*(*A*1) = 0.66 since the EI for the values are

(8) $$\begin{array}{c} I_{10}=0;I_{11}=1;I_{12}=0. \end{array}$$

For surgery, the EI is *I*(*A*2) = 0.79 because

(9) $$\begin{array}{c} I_{20}=1;I_{21}=0;I_{22}=0.9183. \end{array}$$

For hygiene, we have *I*(*A*3) = 0.54 since

(10) $$\begin{array}{c} I_{30}=0;I_{31}=0.8811;I_{32}=0.0. \end{array}$$

Regarding the qualification of the personnel *I*(*A*_4_) = 0.81 given that

(11) $$\begin{array}{c} I_{40}=0;I_{41}=0. \end{array}$$

Figure 5 is the DT it generates.

The corresponding DT appears in Figure 6.

See Table 8 below for the inclusion in the analysis of staff qualification. The worst hospital is between 6 and 5; the best two are followed by 1.

Then, the complete DT of the problem is obtained, see Figure 7.

### 3.4. A Study of Environmental Conditions in Homes: A Campaign against the Transmitting Agent of Dengue

A study was carried out in 22.422 dwellings to establish whether they had good conditions (they were not prone to mosquito outbreaks) or bad conditions. Homeownership was considered as the VR, and they used as SVs:

- Highest educational level of one of the family members
- Location
- C is house in a city
- D is apartment in a multifamily building
- M is a room in a condominium
- S is housing in a semiurban area
- U is urban housing
- V is housing in a village

This DT leads us to detect that:

Those classified as middle-level students differentiate between type n S-U-D-V dwellings (which do not differ from each other) and those of type C.

RETRACTED

The percentages classified as good in the two groups cannot be accepted as similar.

For those who have completed primary school, the same thing happens with M and F.

Those who have graduated have the same behaviour in all types of locations. Homeowners differ from nonowners regardless of the level of schooling or location of their home.

## 4. Conclusion

The impact that is desired to obtain with the project in the application of decision and regression trees as a tool for the prognosis of medical conditions is to take optimal management, taking it as a reference in our research and allowing us to use it as a support to be able to carry out an exhaustive and highly comparative analysis of the analysed data and how the algorithms internally carry out their functions and different analysis methods. Results obtained in this study allow us to focus the campaign to eliminate outbreaks and make propaganda aimed at nonuniversity students without property.

## Figures and Tables

**Figure 1:** Diagram of the selection process, accumulation, and processing of data.

**Figure 2:** A decision tree for investment in new equipment when the old one breaks.

**Figure 3:** Decision tree of the behaviour of the total success of emergency surgery cases.

**Figure 4:** Decision tree of psoriasis patients treated with a placebo ointment.

**Figure 5:** Decision tree of the hygiene analysis in the audit of 6 surgical hospitals. The analysis of surgery leads us to Table 7.

**Figure 6:** Decision tree of the analysis when including surgery together with hygiene in the audit of 6 surgical hospitals.

**Figure 7:** Decision tree of the analysis by including personnel qualification and surgery and hygiene in the audit of 6 surgical hospitals.

**Table 1:** Equivalence of terms between statistics and artificial intelligence.

Statistics	Artificial intelligence
Model	Network
Observations, individuals, and items	Examples of patterns (features, inputs, and outputs)
Independent, explanatory variables, and regressors	Inputs
Dependent variables, responses, and returning	Outputs (outputs and targets)
Waste	Mistakes
Parameters	Weights and synaptic coefficient (weights and synapsis)
Estimation and prediction	Training and learning (training and learning)
Fit criteria	Error function and cost
Regression. Discrimination	Supervised learning
Classification	Unsupervised learning

**Table 2:** Results in the study of successes in emergency surgery.

Atributo	Characteristics	Decision	Attribute
Nivel de la urgencia (*A*_1_)	High	Medium	Under
Estado del salón (*A*_2_)	Okay	Regular	—
Nivel de preparación del personal en la guardia quirúrgica			
Cirujano (*A*_3_)	Optimum	Acceptable	
Personal auxiliary (*A*_4_)	Optimum	Acceptable	
Condiciones físicas del enfermo (*A*5)	Okay	Regular	Bad

RETRACTED

**Table 3:** Entropy gain of attributes.

Attribute	Gain
Urgency level (A1)	0.2728
Hall status (A2)	0
Level of preparation of the personnel in the surgical ward	0.015
Surgeon (A3)	0.226
Auxiliary staff (A4)	0.015

**Table 4:** Results of treatment with a placebo ointment of psoriasis.

			Considered cured		
Cell	Improved	Did not improve	Relapsed	They did not relapse	Total
Red	53	127	0	0	180
Blue	0	62	54	64	180
Total	53	189	54	64	360

**Table 5:** Results of the audit of 6 surgical hospitals.

Hospital	Category	Primary assistance	Surgery	Hygiene	Staff qualification
Hospital-1	NC	M	B.	R	R
Hospital-2	C	M	B.	M	B
Hospital-3	NC	M	R	B.	R
Hospital-4	NC	B	M	M	R
Hospital-5	C	M	B.	M	R
Hospital-6	C	MM	MM	M	R

**Table 6:** Results of the hygiene analysis in the audit of 6 surgical hospitals.

Good hygiene	Primary assistance	Surgery	Hygiene	Staff qualification	Category
Hospital 3 regular hygiene	M	R	B.	R	NC
Hospital 1 poor hygiene	M	B.	R	R	NC
Hospital 2	M	B.	M	B.	C
Hospital 4	B.	M	M	R	NC
Hospital 5	M	B.	M	R	C
Hospital 6	MM	MM	M	R	C

**Table 7:** Results of the analysis when including surgery together with hygiene in the audit of 6 surgical hospitals.

Good surgery	Primary assistance	Surgery	Hygiene	Staff rating	Category
Hospital 2	M	B.	M	b.	C
Bad surgery					
Hospital 5	M	B.	M	R	C
Surgery very bad					
Hospital 4	B.	M	M	R	NC
Hospital 6	MM	MM	M	R	C

**Table 8:** Results of the analysis when including personnel qualification and surgery and hygiene in the audit of 6 surgical hospitals.

Staff rating	Primary assistance	Surgery	Hygiene	Staff qualification	Category
Good					
Hospital 2	M	B.	M	B.	C
Regular staff qualification					
Hospital 5	M	B.	M	R	C

## Data Availability

The data used to support the findings of this study are included within the article.
